RETRACTED

# miR-34a inhibits melanoma growth by targeting ZEB1

**DOI:** 10.18632/aging.203114

**Published:** 2021-06-08

**Authors:** Yazhen Xu, Bingyu Guo, Xiaoyan Liu, Kai Tao

**Affiliations:** 1 Reconstructive and Plastic Surgery, General Hospital of Northern Theater Command, Shenyang, P.R. China

**Keywords:** miR-34a, melanoma, ZEB1, proliferation, migration

## Abstract

Melanoma is a highly lethal cutaneous cancer with the tendency for early invasion and metastasis. Integrated miRNA transcriptome sequence analysis of human melanoma tumors and adjacent control tissues identified 17 miRNAs differentially expressed in melanoma tissues: let-7a-5p, let-7b-5p, let-7c, miR-374a-3p, miR-100-5p, miR-7, miR-195, miR-1908, miR-214, miR-221, miR-199a-5p, miR-21, miR-18, miR-34a, miR-199a-3p, miR-92a and miR-106b. Among these, miR-34a was most significantly down-regulated in melanoma tissues, and its expression correlated with TNM melanoma stage. miR-34a overexpression inhibited expression and activity of the transcription factor ZEB1, resulting in decreased proliferation and migration of melanoma cells. Moreover, miR-34a overexpression inhibited ZEB1 expression and melanoma tumor growth *in vivo*, in a melanoma nude mouse model. Together, these findings demonstrate that miR-34a inhibits melanoma growth by targeting the proto-oncogene ZEB1 and suggest the miR-34a -ZEB1 axis may serve as a novel target for melanoma treatment.

## INTRODUCTION

Melanoma is a highly lethal cancer that occurs predominantly in skin tissues, but also in mucous membranes and eyes. Since melanoma is caused by many factors, including environmental and genetic factors, it is important to identify the genes and their regulatory mechanisms involved in melanoma pathogenesis.

MicroRNAs (miRNAs) are small endogenous non-coding RNAs with 18~24 nt in length. By binding to the 3’-untranslated region (UTR) of target mRNAs, miRNAs regulate gene expression at post-transcriptional level [1–3]. MiRNAs have been implicated in a wide range of cell functions, such as proliferation, migration, apoptosis and differentiation. Dysregulation of miRNAs has been observed in many malignant tumors and plays an important role in tumor development [4]. Recent studies have suggested that miRNAs also regulate proliferation and differentiation of cancer stem cells. According to their role in tumor development, miRNAs can be divided into two groups: Oncogenic miRNAs that are upregulated in cancer cells and promote carcinogenesis by inhibiting tumor suppressor genes, and tumor suppressor miRNAs that prevent cancer development by inhibiting expression of proto-oncogenes.

In melanoma, expression of several members of the miR-let-7 family is decreased; miR-let-7a inhibits expression of the proto-oncogene NRAS [5]. MiR-193b is also down-regulated in melanoma, resulting in the increased expression of Cyclin D1 and proliferation of melanoma cells [6]. In addition, increased expression of miR-205 inhibits melanoma growth [7, 8]. These studies indicate that miRNAs regulate multiple targets that affect different biological functions of melanoma cells. miR-34a is a tumor suppressor miRNA that suppresses tumor development in multiple carcinomas including colon, prostate, and pancreatic cancer. Recent studies have shown that miR-34a also exhibits tumor suppressor characteristics in a variety of cancer stem cells, but its role in melanoma remains to be elucidated.

RETRACTED

Zinc finger E-box binding homeobox 1 (ZEB1) is a transcriptional inhibitor of E-cadherin. By binding to the E-box region of E-cadherin promoter, ZEB1 inhibits E-cadherin expression, resulting in decreased cell adhesion, and increased cell proliferation and metastasis. In this study, we show that miR-34a inhibits occurrence and development of melanoma by inhibiting the ZEB1 expression, indicating that miR-34a might serve as a novel therapeutic target in melanoma.

## RESULTS

### miR-34a targets ZEB1 in melanoma

To elucidate the role of miRNAs in melanoma, we compared expression profiles of miRNAs in melanoma tissues and adjacent tissues by miRNA microarray. The results showed that the expression of let-7a-5p (Flod=4.39), let-7b-5p (Flod=4.45), let-7c (Flod=4.77), miR-374a-3p (Flod=4.62), miR-100-5p (Flod=3.82), miR-7 (Flod=2.94), miR-195 (Flod=2.54), miR-1908 (Flod=2.38), miR-214 (Flod=2.56), miR-29 (Flod=3.96), miR-17 (Flod=2.33), miR-221 (Flod=2.55), miR-199a-5p (Flod=2.41), miR-21 (Flod=2.08), miR-18 (Flod=2.54), miR-222 (Flod=2.86), miR-34a (Flod=23.11), miR-199a-3p (Flod=3.17), miR-19 (2.06), miR-92a (Flod=2.32), and miR-106b (Flod=3.63) differed between melanoma and adjacent control tissues. Among the above miRNAs, miR-34a was down-regulated most significantly in melanoma tissues (Figure 1A). The microarray results were confirmed by real-time PCR; the expression of miR-34a was significantly downregulated in 30 collected melanoma tissues (Figure 1B). The miR-34a expression correlated with TNM stage of melanoma, but not with age and sex (Table 1). miR-34a can bind to 3'UTR regions of multiple proteins. Targetscan and MIRDB analyses indicated that miR-34a could bind to the transcription factor ZEB1 (Figure 1C). Real-time PCR showed that the ZEB1 expression in melanoma tissues was significantly higher than in adjacent tissues (Figure 1D). The expression of miR-34a negatively correlated with the expression of ZEB1 (Figure 1E). Luciferase reporter gene assay showed that miR-34a could suppress ZEB1 activity by targeting ZEB1. However, when the binding site of ZEB1 for miR-34a was mutated, miR-34a did not inhibit the ZEB1 activity (Figure 1F).

RETRACTED

**Figure 1:** **miR-34a targets ZEB1 in melanoma.** (**A**) Microarray analysis of differentially expressed miRNAs in melanoma tissues and adjacent tissues. (**B**) Real-time PCR analysis of miR-34a in melanoma and adjacent tissues (mean ± SEM; ** P< 0.05). (**C**) Targetscan and MIRDB analysis indicating that miR-34a binds to the 3'UTR region of ZEB1. (**D**) Real-time PCR analysis of ZEB1 in melanoma and adjacent tissues (mean ± SEM; ** P< 0.05). (**E**) Negative correlation between miR-34a and ZEB1 expression in melanoma. (**F**) Luciferase reporter assay demonstrating that miR-34a inhibits ZEB1 WT activity, but not ZEB1 MUT activity; ** P< 0.05 vs. control.

**Table 1:** The relationship between miR-34a expression and stages of melanoma.

**Variables**	**Description**	**No. of patient**	**miR-34a expression**		**χ^2^**	***P* value**
			**Low**	**High**		
Gender	Male	19	10	11	0.344	0.558
	Female	11	7	9		
Age(years)	<60	12	7	5	0.023	0.880
	≥60	18	10	8		
Family history	Yes	5	3	2	0.027	0.869
	No	25	14	11		
TNM grade	I	7	1	1	8.285	0.016**
	II	15	9	14		
	III	8	7	5		

T, primary tumor; N, regional lymph nodes; M, metastasis. **, *P*<0.05.

### miR-34a inhibits proliferation and migration of melanoma cells

miR-34a was up-regulated and down-regulated in A375 and A875 cells, respectively. Our results showed that increased miR-34a expression inhibited ZEB1 mRNA and protein levels, and miR-34a suppression increased the ZEB1 levels (Figure 2A–2D). Cell proliferation analyzed by MTT assay was decreased in cells overexpressing miR-34a, and increased in cells with suppressed miR-34a expression (Figure 2E, 2F). Transwell assay showed that migration of A375 and A875 cells was significantly inhibited by miR-34a up-regulation, and increased by miR-34a down-regulation (Figure 2G–2J).

**Figure 2:** **miR-34a inhibits proliferation and migration of melanoma cells.** (**A**, **B**) Western blotting and real-time PCR analysis of miR-34a and ZEB1 in cells overexpressing miR-34a;** P< 0.05 vs. control. (**C**, **D**) Western blotting and real-time PCR analysis of miR-34a and ZEB1 in cells with down-regulated miR-34a expression;** P< 0.05 vs. control. (**E**, **F**) MTT cell proliferation assay in A375 and A875 cells transfected with miR-34a mimic/inhibitor (mean ± SEM; ** P< 0.05 vs. control). (**G**–**J**) Transwell cell migration assay in A375 and A875 cells transfected with miR-34a mimic/inhibitor (mean ± SEM; ** P< 0.05 vs. control).

### miR-34a inhibits proliferation and migration of melanoma cells by targeting ZEB1

To determine whether miR-34a inhibits melanoma cell proliferation and migration through targeting ZEB1, we constructed A375 cells with increased and decreased miR-34a and ZEB1 expression. The promoting effect of miR-34a suppression on cell proliferation and migration could be attenuated by ZEB1 overexpression. The inhibitory effect of miR-34a upregulation on cell proliferation and migration was restored by ZEB1 suppression (Figure 3A–3C). Western blot and real-time PCR showed that the inhibitory effect of miR-34a on ZEB1 expression could be restored by ZEB1 transfection (Figure 3D, 3E).

RETRACTED

**Figure 3:** **miR-34a inhibits proliferation and migration of melanoma cells by targeting ZEB1.** (**A**) MTT cell proliferation assay in A375 cells with increased and suppressed miR-34a expression, and transfected with ZEB1 or ZEB1 siRNA (mean ± SEM; ** P< 0.05 vs. control, ##*P*< 0.05 vs. miR-34a group). (**B**) Transwell migration assay in A375 cells overexpressing miR-34a and transfected with ZEB1 (mean ± SEM; ** P< 0.05 vs. control, ##*P*< 0.05 vs. miR-34a group). (**C**) Transwell migration assay of A375 cells with downregulated miR-34a and transfected with si-ZEB1 (mean ± SEM. ** P< 0.05 vs. control, ##*P*< 0.05 vs. miR-34a inhibitor group. (**D**) Western blotting and real-time PCR analysis of miR-34a and ZEB1 in A375 cells transfected with ZEB1 and overexpressing miR-34a (mean ± SEM; ** P< 0.05 vs. control, ##*P*< 0.05 vs. miR-34a group). (**E**) Western blotting and real-time PCR analysis of miR-34a and ZEB1 in A375 cells with downregulated miR-34a and transfected with si-ZEB1 (mean ± SEM; ** P< 0.05 vs. control, ##*P*< 0.05 vs. miR-34a inhibitor group).

### miR-34a inhibits *in vivo* melanoma growth by targeting ZEB1

Our *in vivo* data using a melanoma nude mouse model showed that miR-34a significantly inhibited the tumor volume and weight; however, when co-transfected with ZEB1, the tumor volume and weight were close to the control group (Figure 4A, 4B). In addition, miR-34a significantly inhibited tumor ZEB1 mRNA and protein levels; however, when co-transfected with ZEB1, the ZEB1 expression was close to the control group (Figure 4C–4E).

**Figure 4:** **miR-34a inhibits *in vivo* growth of melanoma by targeting ZEB1.** (**A**, **B**) Tumor volume and weight in nude mice 28 days after injection with miR-34a and ZEB1 transfection (mean ± SEM; ** P< 0.05 vs. control, ##*P*< 0.05 vs. miR-34a group). (**C**) Immunofluorescence staining of ZEB1 showing increased ZEB1 expression in control group than in miR-34a group, and in miR-34a+ZEB1 group than in miR-34a group (** P< 0.05 vs. control, ##*P*< 0.05 vs. miR-34a group). (**D**, **E**) miR-34a could significantly down regulate ZEB1 expression. ZEB1 transfection attenuated the effect of miR-34a. Data are shown as mean ± SEM. ** P< 0.05 vs. control, ##*P*< 0.05 vs. miR-34a group.

RETRACTED

## DISCUSSION

miR-34a is a tumor suppressor miRNA that has been widely studied in recent years [9, 10]. miR-34a exhibits an abnormal expression in many tumor types. In gliomas, miR-34a expression decreases with increasing clinical grade, which closely correlates with decreased survival time [11]. In colon cancer, the miR-34a expression decreases with the development or metastases [9, 12]. In a mouse model, miR-34a mimic given by tail vein injection or subcutaneous injection reduces distant metastases of osteosarcoma, breast cancer, lung cancer, liver cancer and other tumors [9, 13]. Exogenous miR-34a inhibitor promotes lung metastasis of prostate cancer. miR-34a inhibits uveal melanoma cell proliferation and migration through downregulation of c-Met [14]. miR-34a inhibits melanoma tumor growth by directly targeting the FLOT2 gene [15]. By analyzing 30 pairs of melanoma tissues, we found that many miRNAs were abnormally expressed in melanoma, and that miR-34a was the most significantly down-regulated miRNA in melanoma. In addition, our data showed that the miR-34a expression correlated with the melanoma stage.

The transcription factor ZEB1 is highly expressed in a variety of human cancers, including lung cancer, hepatocellular carcinoma, and breast cancer. Since ZEB1 suppression reduces proliferation and metastasis of cancer cells [16], it represents a potential therapeutic target. In prostate cancer, ZEB1 overexpression has become an important marker for metastasis evaluation [17]. In clear cell renal cell carcinoma, ZEB1 promotes tumorigenesis [18]. In endometrial carcinoma, ZEB1 reduces expression of E-cadherin, resulting in increased invasion and cancer cell migration [19]. In addition, ZEB1 promotes malignant progression of breast cancer and makes breast cancer cells show the characteristics of stromal cells [20]. ZEB1 has been considered as an important EMT related transcription factor, which controls the induction and maintenance of a variety of mesenchymal characteristics. Furthermore, a recent study has indicated that down-regulation of ZEB1 reduces invasive ability of the highly invasive melanoma A375 cells [21].

Our data show that ZEB1 is significantly up-regulated in melanoma tissues and its expression negatively correlates with the miR-34a expression. By targeting the 3'UTR region of ZEB1, miR-34a suppresses the expression and activity of ZEB1. Suppression of ZEB1 by miR-34a results in decreased proliferation and migration of melanoma cells. In addition, our results demonstrate that miR-34a suppresses the ZEB1 expression and inhibits melanoma tumor growth *in vivo*, in a nude mouse melanoma model. These findings identify miR-34a as a potential novel target for the melanoma treatment.

RETRACTED

## MATERIALS AND METHODS

### Tissue samples and cell lines

From January 2012 to December 2018, 30 cases of melanoma tissues were surgically removed in the General Hospital of Northern Theater Command; adjacent tissues were taken as controls. All experiments were approved by the ethics committee of the General Hospital of Northern Theater Command, and all subjects signed written informed consent.

Fibroblasts, A375, and A875 cells were cultured in DMEM / F12 medium (Gibco) containing 10% fetal bovine serum (FBS; Gibco) at 37° C, 5% CO2 and saturated humidity.

### miRNA microarray analysis

MiRNA microarray technology was developed by Duke University gene chip center. The chip contains 1810 miRNA probes from Ambion and Invitrogen. RNA labeling and microarray incubation were performed according to miRCURY LNA miRNA microarray kit. Axon GenePix Scanner (GenePix 4000B) was used to analyze the chip data. Dye-swap was used to design biological repetition. The chip data were analyzed by GeneSpring GX 11.0 software. The Lowess normalization method was used to filter the parameters whose original value was less than 10. The comparison between groups was taken as Flod > 2, P < 0.05.

### Cell transfection

ZEB1, si-ZEB1, miR-34a mimic, miR-34a inhibitor and their negative controls were dissolved in DEPC water at the recommended concentrations. Cells were transfected using Lipofectamine 2000 with the following sequences: miR-34a mimic (sense, 5’-UGG CAG UGU CUU AGC UGG UUG UU-3’; antisense 5’-CAA CCA GCU AAG ACA CUG CGA AA-3’), control (sense, 5’-UUC UCC GAA CGU GUC ACG UTT-3’; antisense, 5’-ACG UGA CAC GUU CGG AGA ATT-3’), miR-34a inhibitor (5’-ACA ACC AGC UAA GAC ACU GCC A-3’), and inhibitor control (5’-CAG UAC UUU UGU GUA GUA CAA-3’).

### MTT assay

Transfected cells were suspended at a density of 1×10^3^ cells / ml, transferred into 96 well plates (100 μL/well; 3 wells per group), and incubated in 37° C incubator. At 0, 12, 24, 36 and 48 h, 5 μL of MTT solution was added into each well, and the plate was incubated at 37° C for 4 h. The absorbance was measured at 490 nm.

### Transwell assay

200 μL of 1 × 10^5^ cells / ml single cell suspension was added into the upper chamber of Transwell chamber, and 600 μL of DMEM / F12 complete medium containing 10% FBS was added into the lower chamber of Transwell chamber. After 24 h incubation at 37° C, medium in the upper chamber was discarded, the Transwell chamber was taken out, and the remaining cells in the upper chamber were wiped with cotton swabs. The cells were fixed by 4 % paraformaldehyde, stained with 0.4 % trypan blue and observed by inverted light microscope.

RETRACTED

### Quantitative real-time PCR

RNA was extracted using Trizol, and real-time PCR was carried out according to the manufacturer’s instructions using the following conditions: 95° C, 10 min; 95° C, 15 s, 60° C, 60 s, 40 cycles; 72° C, 10 min; each experiment was repeated three times. The results were calculated by 2 ^-ΔΔCT^ and expressed by relative quantitative method. The expression of miR-34a was detected with Stem-Loop RT-PCR assay as reported [22, 23], and all reactions were carried out as described previously [24]. The primer sequences are shown in Table 2.

**Table 2:** Primer sequences.

**Name**	**Forward primer(5'->3')**	**Reverse primer(5'->3')**
miR-34a	TGGCAGTGTCTTAGCTGGTTGT	
U6	CGCTTCGGCAGCACATATACTAAAATTGGAAC	
ZEB1	CAATGATCAGCCTCAATCTGCA	CCATTGGTGGTTGATCCCA
GAPDH	GCACCGTCAAGGCTGAGAAC	TGGTGAAGACGCCAGTGGA

### Western blot analyses

Collected tissues or cells were lysed by RIPA buffer. BCA protein concentration assay kit was used to determine the protein concentration. Proteins were separated by SDS-PAGE electrophoresis and transferred to PVDF membranes. After blocking in 5% skimmed milk, the membranes were incubated with specific antibodies: ZEB1 (sc-515797) and GAPDH (sc-365062)(Santa Cruz).

### Dual luciferase reporter assay

The 3’-UTR fragments of ZEB1 WT (F:5'GATCCTTCTGGAGAGGTCAGAGTTGACAAGCTTG'3, ZEB1 -3’UTR-R:5'AATTCAAGCTTGTCAACTCTGACCTCTCCAGAAG'3) and ZEB1 MUT (mutant miR-34a-binding sites, F:5'GATCCTTCTGGAGAGGTGTCTCTTGACAAGCTTG'3, ZEB1-3’UTR-R:5'AATTCAAGCTTGTCAACTCTGACCTCTCCAGAAG'3) were constructed by Changsha Yingrun Co., Ltd., and inserted into the pMIR-REPORT miRNA Expression Reporter vector (Ambion; Thermo Fisher Scientific); they were labeled as pMIR-ZEB1-3’-UTR. Cells were plated into 24-well plates 1 night before transfection. miR-34a (20 nM, 5’-UGGCAGUGUGGU UAGCUGGUUGU-3’) or miR-NC (20 Nm, 5’-CAGUACUUUUGUGUAGUACAA-3’) were co-transfected with pMIR-ZEB1-3’-UTR (100 ng) into cells using Lipofectamine 2000 reagent according to the manufacturer’s recommendations. Transfected cells were collected after 48 hours of incubation at 37° C and then luciferase activity was measured using a dual-luciferase reporter assay system (Promega Corporation, Fitchburg, WI, USA) in accordance with the manufacturer’s instructions. Firefly luciferase activity was normalized to that of Renilla luciferase [25].

### Establishment of nude mice melanoma model

Eighteen nude mice were divided into three groups (n=6): Control miRNA (control group), miR-34a overexpression group, and miR-34a+ZEB1 group. Five-week-old BALB/c male nude mice were purchased from Beijing Laboratory Animal Research Center (Beijing, China). Mice were housed in conditions in accordance with the guidelines of experimental animal center of General Hospital of Northern Theater Command. Tumor volumes were measured every four days with a digital caliper following the formula: Volume = 0.5 × (width^2^ × length). Twenty-eight days post injection, mice were sacrificed using carbon dioxide inhalation, and tumors were resected, weighed, and analyzed for ZEB1 expression.

RETRACTED

### Immunofluorescence staining

Five consecutive sections of each tumor tissue were deparaffinized in xylene. After rehydration by a series of graded alcohols, 0.01 M sodium citrate (pH 6.0) was used to perform antigen retrieval. After blocking by goat serum (15 min at room temperature), the sections were incubated (12 h, 4° C) with primary antibody, followed by secondary antibody (15 min, 37° C). After washing, the sections were stained with horseradish enzyme-labeled streptavidin and DAB, and counterstained with hematoxylin. Five slices of each section were randomly selected to count ZEB1 positive cells and percentage of positive cells was calculated. Cells with brown particles in cytoplasm were considered as ZEB1 positive cells.

### Statistical analysis

The SPSS17.0 software was used for statistical analysis. Mann Whitney U-test was used to compare the difference of tumor formation in each group; P < 0.05 was considered statistically significant.
